# Analysis on the Impact and Management of Political Education of College Students in the Micro Era Environment

**DOI:** 10.1155/2022/7103268

**Published:** 2022-08-08

**Authors:** Li Li, Wei Li

**Affiliations:** Graduate School, University of Perpetual Help System DALTA, Las Pinas 1740, Philippines

## Abstract

With the rapid development of modern society and the popularization of information equipment, information transmission has broken the time and space constraints, and political education (PE) can be carried out anytime and anywhere. Micro media is the product of the rapid development of science and technology, which has brought us into a new “micro era.” The research on the “micro era” has been the focus of academic attention in recent years. Especially with the popularization of micro media, its influence on people is becoming deeper, making more scholars in academic circles devote themselves to the “micro era” under study. However, while micro media is widely used by college students (CS), it also brings opportunities and challenges. Therefore, it is particularly important to clarify the opportunities and challenges faced by CS' PE under the background of the “micro era” and put forward practical countermeasures. Starting from the actual situation of PE communication in the micro era, this study analyzes the opportunities and challenges brought by the “micro era” to PE of CS through a questionnaire survey. Then, the effective strategies to improve the PE of CS are explored, in order to improve the ideological and political level of CS in the micro era.

## 1. Introduction

College students are the most dynamic and creative group, and the bright future of our country cannot be separated from their hard work [1]. Just as General Secretary Xi said, “The Chinese dream belongs to us, especially to your younger generation. The great rejuvenation of the Chinese nation will become a reality through the relay struggle of the vast number of young people.” CS are the vanguard of the times and the future of the nation, and their future is related to the fate and future of the country [2]. Training and paying attention to their growth is of great practical importance to the realization of our great dream and the construction of our great cause.

With the rapid development of network information technology and the “micro era,” micro things represented by Weibo and WeChat occupy the forefront position of network platforms rapidly with the advantages of diversified content, open platform, and powerful functions [3]. CS have become loyal supporters and promoters of the “micro era,” which has created a “micro whirlwind” on university campuses. Their life, study, and work have permeated the atmosphere of the “micro era” [4].

With the rapid popularization of Microblog and WeChat among CS, various social trends of thought and decadent and backward thoughts are also disseminated to CS through micro media, impacting the mainstream values of our country [5]. Due to their immature mind and lack of social experience, some CS are prone to deviation in value orientation, ideal and belief, and behavioral cognition. Universities must strengthen PE to study the “micro era.” Therefore, this study conducts a questionnaire survey on PE of CS under the background of the “micro era” by studying the current situation of PE in the micro era and analyzes the situation of PE carried out by micro media. Finally, the realization path of CS' PE under the background of the “micro era” is put forward.

This study has the following research significance: first, it has expanded and enriched the research content of PE for CS. Second, it promotes the theoretical innovation of PE in colleges. Third, it deepens the research on PE of CS under the background of the “micro era.” Fourth, it is beneficial to enhance the effectiveness of CS' PE. Fifth, it is conducive to the sound development of the “micro era.” Last, it is conducive to training qualified builders and successors.

This article consists of five main parts: the first part is the introduction, the second part is the state of the art, the third part is the current methodology, the fourth part is the result analysis and discussion, and the last part is the conclusion.

## 2. State of the Art

### 2.1. Constituent Elements of PE Communication

The communication elements of PE constitute the basic framework of the communication system of PE [6]. Understanding the elements of PE communication is beneficial for us to reasonably grasp its internal structure, mechanism of action, and communication process [7]. The components of PE communication mainly include the PE communication subject, PE communication content, PE communication media, PE communication audience, and PE communication environment.

The subject of PE dissemination is not only the sender of PE information but also the guide and manager of PE dissemination [8]. It includes front-line ideological and political teachers, counselors, scholars and experts in PE, and other PE workers. The main body of PE communication plays a leading role in the process of communication [9]. The establishment of communication objectives, the selection of content, the management of the communication process, and the prediction of communication effects are inseparable from the careful management of PE communicators. The knowledge structure and control ability of PE communicators directly affect the process and validity of communication [10]. Solid professional knowledge is conducive to the dissemination of sports information in the tide of sports information pollution, as well as the screening of high-quality sports information. Good regulation ability is beneficial for PE communicators to deal with emergencies flexibly, coordinate various elements, and make reasonable use of communication skills. Therefore, this requires the dissemination of PE to enhance their own ability to check and improve the ideological quality, sound personality quality. At the same time, the psychological law and educational law of the communicator are followed to influence the communicator's management and communication process.

The content of PE communication is PE information [11]. It generally includes five aspects: politics, ideology, legal system, morality, and psychology. The communication content of PE occupies the core position in the process of communication. Due to the special role of PE content, the content is required to be legitimate, reasonable, objective, and scientific [12]. In a particular dissemination process of PE, the content of PE is also required to conform to the objective laws and to match the acceptable degree of the educatee. For primary- and middle-school students, PE information is required to be easy to understand and easy to internalize and absorb. For CS, PE information is required to be objective and profound, theoretical, and enlightening.

The media of PE include classrooms, party congress, the Internet, TV, books, and periodicals [8]. According to different sign forms, it can be divided into electronic media, physical media, and language media. According to norms, it can be divided into formal media and informal media. The media of PE plays an important role in the process of its communication, which is the link connecting other communication elements [13]. Contemporary media are mixed, which requires the disseminators of PE to deeply understand and grasp the media, understand the advantages and disadvantages of various media, and use the media to carry forward the socialist core values.

The dissemination audience of PE is the receiver and host of PE information. No matter from the perspective of PE communication motivation, or from the perspective of testing the effect of communication, the audience is indispensable, and without an audience, communication will have no meaning. In the communication of political education, the communication subject should not only follow the psychological law of the audience but also understand the personality and preference of the audience and pay attention to the object characteristics of the audience. The motivation theory should also be used to stimulate the learning motivation of the audience and enhance the main characteristics of the audience.

The PE communication environment also plays an important role in the operation of the PE communication system. The communication environment of PE includes not only the social and cultural environment of the communication but also the accompanying psychological environment of the communicator and the audience. It also includes the physical environment, such as communication facilities and surrounding buildings. The social and cultural environment and the psychological environment of the subject have a greater impact on the dissemination of PE than the physical environment. The environment has a subtle influence on the subject of transmission, so the PE should pay attention to optimizing the environment.

These elements depend on each other and interact with each other, constituting the dissemination process of PE.  Figure 1 is the communication process of PE. It represents ①the screening and sorting of communication content, ②the selection of media, ③the reception of communication content, ④the feedback information, and ⑤the influence of the environment on the other four elements. As can be seen from the figure, the communication subject of ideological organization education first screens and arranges the communication content and then selects the appropriate communication media to deliver the PE content to the audience. The audience receives the communication content and gives feedback on the communication subject. During this period, the communication environment of PE will affect the psychological state of the communication subject and the link of integrating information, the link of transmitting PE content, and the link of receiving information. Therefore, the communication elements of PE are interrelated and constitute an organic and unified whole.

### 2.2. Overview of the Micro Era

As information media change with each passing day, the micro era marked by the widespread use of new media such as Weibo, WeChat, and mobile apps has arrived [14]. Although the micro age has entered, there is still no unified definition of the micro age in academic circles so far, and the micro age is a relative concept at present [15].

From the perspective of information dissemination, the micro era refers to a new era of real-time and efficient communication based on information digitization technology, using digital communication technology, using audio, video, text, image, and other ways through new, mobile, and convenient display terminals. In terms of media, the micro era refers to the application era represented by WeChat and Weibo. From the perspective of content, the micro era includes micro video, micro audio, micro quotes, micro public welfare, and micro movies. In terms of audience, all the people who use Weibo, WeChat, and mobile apps are called Weimin. Micro citizens can use the media to express their views. From the perspective of life, the micro era is accompanied by the micro psychology, micro habits, and micro communication era.

In the micro era, digital technology and network information technology are booming, we media are rising rapidly, and media are becoming diversified. Contemporary media are numerous in variety and function [16].

In the micro age, information presents the characteristics of popularization, which is mainly manifested in two aspects. On the one hand, in today's society, the development of “we media” is booming, and the entry threshold is low. The main disseminators are civilians, and everyone is an “independent media person.” People can speak freely on “we media,” publish what they think, and record what they see and hear on that day. On the other hand, in the micro age, information is no longer a one-way flow like the traditional TV, but a multi-level and multi-directional flow form. In addition to posting information, people can freely comment, like, and retweet.

The micro era is characterized by open communication [17]. Under the background of the micro era, the communication threshold is low, and an asymmetric interpersonal relationship has been formed on the network media. The micro era is characterized by strong openness in communication. The open environment enables information transmission to form a multi-directional interactive mode, and the openness of “we media” makes the audience actively participate in it.

With the development of network information technology, information transmission transcends the limitation of time and space, and the transmission speed is calculated in seconds, with high speed and efficiency. The instantaneity of communication is a remarkable feature of the micro age [18].

Micro age has spread widely. Due to the characteristics of split-change communication of “we media,” the scope of information dissemination is very wide [19].  Figure 2 is a diagram of the model of the fissionable spread of information, in which one information source can be transmitted to multiple audiences such as ABC (primary transmission). Audience *G* transmits the information to G1 (secondary transmission) through its own understanding, and G1 passes to G2, and G2 spreads until Gn, which forms the fissionable spread. Fragmentation communication enables a single source of information to be transmitted to thousands of audiences, and information diffusion increases exponentially.

## 3. Methodology

“Micro era” is a double-edged sword, which brings both new opportunities and new challenges to PE in colleges. In order to fully understand the new situation of PE in colleges in the “micro era,” this study designed a questionnaire. It is expected to investigate and analyze the opportunities and challenges brought by the “micro era” to PE in colleges and then explore specific coping strategies. In order to better analyze the status quo of PE in colleges in the “micro era,” an anonymous questionnaire survey was carried out on the network. This survey is mainly about the current situation of CS' use of Microblog and WeChat. The survey content is divided into two parts: basic information and questionnaire content. A total of 524 questionnaires have been issued and 524 have been recovered, with an effective recovery rate of 100%.

### 3.1. Analysis of Survey Objects

The first part of the questionnaire is about the basic information of the respondents. There are six questions in total, including gender, school, grade, major, school identity, and political status. In general, by investigating the basic information of CS from different aspects, we can have a comprehensive understanding of the influence of the “micro age” represented by Microblog and WeChat on CS so that the survey results are authentic and reliable.

### 3.2. Analysis of CS' Use of Micro Media

By collecting and sorting out 524 questionnaires, we have a general understanding of the purpose and situation of the use of micro media by CS. According to the survey results, the influence of micro media on CS is analyzed from the following aspects.

In terms of the opening situation, 298 of the 524 CS surveyed have opened micro blog.

WeChat accounts for 56.87%; 156 people have only opened Weibo and 70 people have only opened WeChat, accounting for 29.77% and 13.36%, respectively. Among the respondents, there is no one who does not use Weibo and WeChat (see Figure 3). It can be seen that Weibo and WeChat, as the most popular software at present, have a high popularity rate among young CS. It is favored by the student community.

In terms of using time, the number of people who use micro media for 1–3 hours a day is the largest, accounting for 44.66% (234 people), and the number of people who use more than 5 hours a day is the least, accounting for 8.4%. In terms of the advantages of micro media, the CS who choose rich information, timely updates, convenient login, diversified platform, and strong interaction are the most, accounting for 59.35%, 56.68%, and 51.91%, respectively. 181 people and 166 people chose powerful, easy to operate, cheap, and widespread (see Figure 4). It can be seen that the unique advantages and powerful functions of micro media are very attractive to CS and occupy a lot of time and energy of CS.

In terms of the target and content (see Figures 5 and 6), the preferred target of CS' attention on micro media is classmates and friends (55.73%), Internet celebrities (52.29%), and star idols (48.66%). It was followed by experts and scholars (35.5%), teachers and counselors (29.58%), and official Weibo and official accounts (21.18%). Entertainment gossip (61.64%) and learning materials (57.44%) are the most popular choices for micro media. Employment information (47.33 percent) and current politics news (37.6 percent) followed by life information (29.39 percent) and others (12.6 percent).

As for use, considering that there may be huge differences in the purpose of micro media use by CS, the sixth question is set as a sorting question (see Figure 6). According to the ranking of the specific items in the question, the survey results show that the ranking of expressing opinions is the first, followed by leisure and entertainment, learning cultural knowledge, and making friends and chatting lastly (see Figure 7). It can be seen that the emergence of micro media meets the basic needs of CS and is an important medium for CS to obtain information, relax their mood, and make friends with each other.

In terms of using time, the majority of people choose to use Weibo and WeChat during class, boring period, and waiting periods, accounting for 58.4%, 56.49%, and 49.05% respectively. The second choice is when taking transportation accounting for 41.98% and before going to bed accounting for 30.73%; the number of people who choose other time accounts for only 8.59%. It can be seen that the emergence of micro media can effectively meet the needs of CS in fragmented time, such as receiving information, leisure and entertainment, and releasing pressure, and it has become the urgent need of CS to kill fragmented time.

In terms of the impact of micro media on CS, 32.06% of them think micro media has a great impact on their outlook, life, and cognition, 32.82% of them think it has a general impact, 21.37% of them chose to have a great impact, and only 13.74% of them think micro media has no impact. From the perspective of the influence of micro media peers, 36.83% of students choose their own value orientation, ideology, and other ideas that are greatly influenced by their peers. 26.53% and 18.89% of the students chose to have a great influence and an average influence, while 9.54% and 8.21% of the students chose to have a little influence and no influence, respectively. According to the survey results, most students believe that micro media has brought changes to their life, study, and thoughts. It can be seen that micro media has an important impact on CS beyond doubt.

In terms of identifying micro media information, 27.67% of the students choose to frequently identify, 32.67% choose to occasionally identify, 24.05% of the students choose never to identify the information released by “BIG V,” and 15.65% of the students choose only to browse, but never to identify the message. It can be seen that most of the students surveyed only occasionally or never identify micro media information. However, as a distribution center of information, micro media inevitably generates fake junk information while producing real useful information. CS lacks discrimination in micro media information, which is bound to hinder the development of their discrimination ability.

### 3.3. Analysis of PE through Micro Media

Through the analysis of the questionnaire survey and the collation of the survey results, the following aspects are analyzed for the use of micro media in PE in colleges.

As for the attitude toward using micro media to carry out PE in colleges, 19.66% of students strongly agree, 28.44% agree, and 26.53% generally agree. The proportion of those who moderately disagree and strongly disagree was 12.98% and 12.4% (see Figure 8). The survey results show that CS are relatively supportive of carrying out PE activities on micro media. Therefore, PE in colleges can effectively use micro media to open up new educational spaces, expand teaching scope, and improve its influence.

In terms of the way of contact between CS and teachers and counselors, 302 of the 524 respondents choose to contact through Weibo or WeChat, 99 choose to be relayed by others, 82 choose to contact by phone or text message, and only 44 choose to have face-to-face contact in the office. In terms of the number of times teachers and counselors communicate with students through micro media, 33.02% of the students think a lot, 30.53% think a lot, 21.76% choose occasionally, and 14.68% choose teachers and counselors do not communicate with students through micro media. The survey results show that Weibo and WeChat, as popular software, are the best choice for educators to communicate with CS promptly. This software effectively reduces the estrangement between the two sides of education, shortens the distance between them, and opens a convenient door for orderly PE in universities.

In terms of PE methods, CS, as trend makers of the new era, are at the forefront of the “micro” trend and the most loyal fans of micro media. They are not only keen on micro media but also put forward corresponding demands for teaching methods. When asked which way do you prefer to carry out PE in the “micro era,” 60.88% of students choose micro media teaching, 57.06% choose a social practice, and 39.89% choose classroom teaching (see Figure 9). Therefore, it is not difficult to see that compared with classroom teaching with a relatively fixed learning environment and “infusing” teaching method, micro media teaching with a loose teaching environment and interactive teaching method is more popular among CS. Therefore, PE in colleges should be good at using micro media and organically combine micro media with teaching work to enhance its appeal.

In terms of the use of micro media to carry out PE, when asked “your university often pushes PE information on micro media,” 24.05% of the students choose often, 31.3% choose occasionally, 24.81% choose rarely, and 19.84% choose almost nothing or pay no attention to it. From the effect of paying attention to and browsing PE information of micro media, 25.57% of those choose to pay attention to and browse frequently, 36.26% of those choose occasionally, 24.24% of those choose rarely, and 13.93% of those choose never to pay attention to and browse. Survey data show that PE in colleges still attaches great importance to the use of micro media platforms to carry out work, but CS do not pay much attention to and browse the PE information on micro media. This shows that the use of micro media in PE in colleges needs to be further improved and perfected, and the content and means of communication should be constantly innovated to enhance the interest of teaching, so as to increase CS' attention to it.”

In terms of improving PE in colleges, when asked what aspects of PE need to be strengthened in the “micro era” (multiple choice), the number of people who choose flexible educational methods and educational content in line with students' needs is the largest, accounting for 56.11% and 54.77% of the total number of people, respectively. The second was to strengthen the construction of teaching staff (44.27%), keep pace with the times (36.45%), and build an online teaching platform (32.25%). The last one was to strengthen network supervision (18.13%) and others (9.16%) (see Figure 10). Survey data show that in order to do a good job in PE in colleges under the new situation, it is necessary to constantly break through themselves from the abovementioned aspects, enhance the ability to adapt to and cope with the “micro era,” and improve the quality of teaching.

In terms of the quality of ideological and political teachers in colleges in the “micro era,” 59.16% of students chose teachers with noble moral quality, 58.59% chose teachers who are caring and close to students, 48.85% chose teachers with equal consciousness, 39.12% think teachers should have a solid professional foundation, 28.82% of the students thought that a teacher should have high media skills, and 12.6% thought that a teacher should have good communication skills (see Figure 11). This shows that the arrival of the “micro era” poses a greater challenge to the comprehensive ability of ideological and political teachers. Ideological and political teachers should constantly strengthen their own ability construction from these aspects, improve the comprehensive quality and personality charm, enhance their professional and technological level, and lay a solid foundation for PE in colleges.

## 4. Result Analysis and Discussion

Through the statistical analysis of the survey data, we can see that the “micro era” brings both opportunities and challenges to the PE of CS. Therefore, at present, we must conform to the trend of the times, actively respond to the threat and challenges under the specific background of the times, and effectively put forward the specific path to carry out the PE in the “micro era.”

### 4.1. Adhering to the Combination of Education and Self-Education and Improving the Quality of Education

At the arrival of a brand new “micro era,” it is difficult for CS to have an objective and comprehensive understanding of micro communication, micro information, and other new things due to their own limitations. Therefore, colleges must attach great importance to the education of universities, guide them to view “micro information” in a comprehensive and dialectical way, and correctly evaluate the impact of “micro communication.” Also, we should recognize that education is an external force, and its role can only be played through the active acceptance and internalization of CS. Therefore, the combination of education and self-education is the inevitable choice to improve the quality of CS.

In the “micro era,” anyone can become an information publisher with the help of a wide variety of micro media. For example, teachers can release the latest educational information through WeChat and Weibo. Schools can release real-time campus consultations through official micro media. The release of micro media information does not need to be strictly reviewed, which makes some negative information emerge at the right moment. Sometimes, this information is so mixed up with positive information that it is hard to judge. Therefore, the current PE must include the improvement of CS' ability to identify micro information. First, ideological and political educators should guide CS to set up the identification thinking of a dialectical view of micro media information. Second, colleges should strengthen media literacy education and improve the information discrimination ability of CS.

Under the background of the “micro era,” it is very necessary for CS to use micro media for self-education. Under the background of the “micro era,” micro media provides diversified information that CS can obtain at will, while ideological and political educators and parents are unable to supervise and guide children at all times. Therefore, it is necessary to learn to use “micro media” for self-education to make up for the lack of school education and family education.

### 4.2. Drawing the Advantages of Micro Media to Enhance the Effect of PE

Under the background of the “micro era,” the problems of PE, such as backward content, single presentation, discourse mode, and rigid educational methods and models, are becoming increasingly prominent. Therefore, in order to do a good job in the PE of CS, we must be guided by the problems existing in the PE of CS and widely absorb the advantages of others to make up for their own shortcomings.

We establish an interactive PE model. First of all, ideological and political educators should give full respect to CS in class, encourage students to actively express their opinions and views, and interact with teachers. In daily life, teachers and students can make friends with each other through micro media to realize after-class “one-to-one” interactive tutoring and promote the benign interaction between teachers and students. Second, it is of great significance to realize the interaction between students in the process of PE. Therefore, ideological and political educators should create an atmosphere for students to communicate and interact. For example, teachers can encourage students to have group discussions in class and set up “micro discussion groups” after class to help students communicate in time and share achievements. Finally, it is necessary to realize not only the interaction between teachers and students and students and students but also the interaction between teachers, which is helpful for teachers to share experiences, supervise each other, and jointly improve their teaching level and research ability. Therefore, colleges should hold regular teacher exchange meetings and academic seminars to promote the interaction between teachers. Ideological and political educators can also add friends to each other through micro media to timely interact and communicate in teaching and work.

### 4.3. Innovating the Carrier of PE and Improving the Influence of Education

Under the background of the “micro era,” with the emergence of micro movies, micro theory, micro blog, WeChat, micro public welfare, and other things, the carrier forms of carrying out PE for CS have been greatly enriched. In particular, the popularization of micro media such as Weibo and WeChat among CS provides an opportunity to innovate the carrier of PE for CS.

Strengthening the “micro construction” and further perfecting the “micro carrier” of PE is an important guarantee to play the positive role of “micro carrier” in the current PE of CS. High-quality “micro carrier” can not only attract the attention of CS but also subtly help them form a correct world outlook, outlook on life, and values. On the contrary, without careful management and strict supervision, micro carriers will not only become the distribution center of undesirable opinions and information but also make the information content and form of micro carriers out of touch with The Times. This makes it difficult for the micro carrier to attract the attention of college students, thus affecting the educational function of the micro carrier.

### 4.4. Making Use of Culture and Management to Optimize the Environment of PE

Under the background of the “micro era,” the network environment is unpredictable, the campus cultural environment is more diversified, and the guidance and management of the college students' peer group are more difficult, which makes the environment of carrying out PE of CS more complicated. Therefore, universities and ideological and political educators must strive to find appropriate ways to optimize the PE environment by the power of culture and management.

With the rapid development of Internet technology, the Internet has become an indispensable part of people's life. Especially with the arrival of the “micro era,” people can participate in the discussion of new situations and new problems with the help of the simple operation of micro media. However, due to the rapid and changeable update of information, people grasp the data and information is also in constant change. In addition, the perspective of each person is affected by factors such as individual living environment and education level. Therefore, the audience will form diverse and rapidly changing online public opinions on the same event or issue. Moreover, some false information, vulgar information, bad speech, and other information flooded the network, which to some extent worsened the PE environment of CS. Therefore, on the one hand, colleges should strictly observe the import and export of information and put an end to the emergence of bad information and false information on the network. On the other hand, we should actively guide public opinion in the right direction of development, achieve the combination of “blocking” and “thinning,” and constantly optimize the network environment of college students' PE.

The network public opinion environment of people's PE in the “micro era” is changing rapidly, sometimes the public opinion will develop in the right direction, and sometimes it will develop in the negative direction. Therefore, ideological and political educators in universities should pay close attention to the trend of public opinion, guide CS to identify the correct direction of public opinion, and purify the network environment so that CS can actively transfer positive energy in the network life, away from bad information.

## 5. Conclusion

The “micro era” is rolling in, and micro media such as micro blog and WeChat have become important communication channels and communication platforms in today's society. Micro media is like a double-edged sword, which brings many opportunities and challenges to PE in colleges. Under the current background, the PE of CS has become more complex and difficult. Due to the impact of foreign culture and the lack of attention of CS to PE, PE in colleges lack effect. Therefore, how to give full play to the advantages of the “micro era” and make good countermeasures against the new problems and situations is of great practical significance to the development of PE in colleges. In view of this, based on the current situation of PE communication in the micro era, this study investigates and studies the PE of CS under the background of the “micro era” and analyzes the situation of PE by using micro media. Finally, this study puts forward the realization path of CS' PE under the background of the “micro era,” focusing on the combination of education and self-education, changing the way of discourse, improving educational methods, innovating the carrier of PE, and strengthening cultural publicity and management. However, because “micro era” is an emerging issue in the current research, the definition of “micro era” in the academic community has not been finalized, and the author's academic level and scientific research ability are limited, and there are still some deficiencies in the research. I hope to be criticized and corrected by experts and scholars.

## Figures and Tables

**Figure 1:** PE dissemination process diagram.

**Figure 2:** Pattern diagram of information cracking propagation.

**Figure 3:** Proportion of opening micro blog and WeChat.

**Figure 4:** Distribution of advantages of micro media.

**Figure 5:** Proportion of the object of attention.

**Figure 6:** Proportion of attention to content.

**Figure 7:** Proportion of purposes of using micro media.

**Figure 8:** Proportion of attitudes towards using micro media for PE in colleges.

**Figure 9:** Proportion of PE mode selection.

**Figure 10:** Proportion diagram of PE in colleges in the micro era.

**Figure 11:** Proportion diagram of political teachers' qualities in the micro era.

## Data Availability

The labeled dataset used to support the findings of this study is available from the corresponding author upon request.

## References

[1] Bae H., Kerr D. C. R. (2020). Marijuana use trends among college students in states with and without legalization of recreational use: initial and longer‐term changes from 2008 to 2018. *Addiction*.

[2] Johnston H. (2019). The elephant in the room: youth, cognition, and student groups in mass social movements. *Societies*.

[3] Cheng Y. (2020). The social-mediated crisis communication research: revisiting dialogue between organizations and publics in crises of China. *Public Relations Review*.

[4] Le H., Guanzhong W. (2020). Research on strategies to improve the media literacy of college students on the platform of micro media in the new era. *The Theory and Practice of Innovation and Entrepreneurship*.

[5] Ji Z. (2020). Exploration and application of micro-project learning in SCM classroom teaching reform. *International Journal of Social Science and Education Research*.

[6] Yu Y. (2022). On the ideological and political education of college students in the new media era. *Open Journal of Social Sciences*.

[7] Yi Y., Dan W. (2020). The realization of ideological and political education in college English based on cultural confidence. *Creative Education*.

[8] Li F., Fu H. (2020). Study on college English teaching based on the concept of ideological and political education in all courses. *Creative Education*.

[9] Xia Y. (2021). Big data based research on the management system framework of ideological and political education in colleges and universities. *Journal of Intelligent and Fuzzy Systems*.

[10] Xiaoyang H., Junzhi Z., Jingyuan F., Xiuxia Z. (2021). Effectiveness of ideological and political education reform in universities based on data mining artificial intelligence technology. *Journal of Intelligent and Fuzzy Systems*.

[11] Yu X., Dong G. (2021). On the ideological and political education of college students in the new media era. *International Journal of Social Science and Education Research*.

[12] Zhou P. (2020). Innovative research on ideological and political education in colleges by improving the effectiveness. *International Journal of Social Science and Education Research*.

[13] Wang Q., Zhou H., Wang P. (2020). Application value of magnetic resonance hydrography of the inner ear in cochlear implantation. *Revista da Associação Médica Brasileira*.

[14] Huang Y., Miao W. (2021). Re-domesticating social media when it becomes disruptive: evidence from China’s “super app” WeChat. *Mobile Media and Communication*.

[15] Lin L., Jiang A., Zheng Y., Wang J., Wang M (2021). New media platform’s understanding of Chinese social workers’ anti-epidemic actions: an analysis of network public opinion based on COVID-19. *Social Work in Public Health*.

[16] Wang L., Situ S., Rainey J. J. (2021). Using weibo and wechat social media channels to assess public awareness and practices related to antimicrobial resistance, China, 2019. *BMC Public Health*.

[17] Qu Y. (2020). Engaging publics in the mobile era: a study of Chinese charitable foundations’ use of wechat. *Public Relations Review*.

[18] Wang D., Yang L., Yue D. (2019). Macrophage-derived CCL22 promotes an immunosuppressive tumor microenvironment via IL-8 in malignant pleural effusion. *Cancer Letters*.

[19] Wang Y. (2020). Analysis on the construction of ideological and political education system for college students based on mobile artificial intelligence terminal. *Soft Computing*.

